# Machine Learning Hybrid Model for the Prediction of Chronic Kidney Disease

**DOI:** 10.1155/2023/9266889

**Published:** 2023-03-14

**Authors:** Hira Khalid, Ajab Khan, Muhammad Zahid Khan, Gulzar Mehmood, Muhammad Shuaib Qureshi

**Affiliations:** ^1^Department of Information Technology, Abbottabad University of Science and Technology, Havelian 22500, Abbottabad, Pakistan; ^2^Department of Computer Science and I.T, Network Systems and Security Research Group, University of Malakand, Chakdara 18800, Khyber Pakhtunkhwa, Pakistan; ^3^Department of Computer Science, IQRA National University, Swat Campus 19220, Peshawar, Pakistan; ^4^Department of Computer Science, School of Arts and Sciences, University of Central Asia, Bishkek, Kyrgyzstan

## Abstract

To diagnose an illness in healthcare, doctors typically conduct physical exams and review the patient's medical history, followed by diagnostic tests and procedures to determine the underlying cause of symptoms. Chronic kidney disease (CKD) is currently the leading cause of death, with a rapidly increasing number of patients, resulting in 1.7 million deaths annually. While various diagnostic methods are available, this study utilizes machine learning due to its high accuracy. In this study, we have used the hybrid technique to build our proposed model. In our proposed model, we have used the Pearson correlation for feature selection. In the first step, the best models were selected on the basis of critical literature analysis. In the second step, the combination of these models is used in our proposed hybrid model. Gaussian Naïve Bayes, gradient boosting, and decision tree classifier are used as a base classifier, and the random forest classifier is used as a meta-classifier in the proposed hybrid model. The objective of this study is to evaluate the best machine learning classification techniques and identify the best-used machine learning classifier in terms of accuracy. This provides a solution for overfitting and achieves the highest accuracy. It also highlights some of the challenges that affect the result of better performance. In this study, we critically review the existing available machine learning classification techniques. We evaluate in terms of accuracy, and a comprehensive analytical evaluation of the related work is presented with a tabular system. In implementation, we have used the top four models and built a hybrid model using UCI chronic kidney disease dataset for prediction. Gradient boosting achieves around 99% accuracy, random forest achieves 98%, decision tree classifier achieves 96% accuracy, and our proposed hybrid model performs best getting 100% accuracy on the same dataset. Some of the main machine learning algorithms used to predict the occurrence of CKD are Naïve Bayes, decision tree, K-nearest neighbor, random forest, support vector machine, LDA, GB, and neural network. In this study, we apply GB (gradient boosting), Gaussian Naïve Bayes, and decision tree along with random forest on the same set of features and compare the accuracy score.

## 1. Introduction

Nowadays, chronic kidney disease (CKD) is a rapidly growing disease, and millions of people die due to lack of timely affordable treatment. Chronic kidney disease patients belong to low-class and middle-classincome-generating countries [1, 2].

In 2013, about one million people died due to chronic kidney disease [3]. The developing world suffers more from the chronic kidney disease, and low to average income countries contain a total of 387.5 million CKD patients where 177.4 million patients are male and 210.1 million patients are female [4]. These figures show that a large number of people in developing countries suffer from chronic kidney disease, and this ratio is increasing day by day. A lot of work has been done for the early diagnosis of chronic kidney disease so that the disease could be treated at an early stage. In this article, we are focusing on machine learning prediction models for chronic kidney disease and giving importance to accuracy.

Chronic kidney disease is a common type of kidney disease that occurs when both kidneys are damaged, and the CKD patients suffer from this condition for a long term. Here, the term kidney damage means any kidney condition that can cause improper functioning of the kidney. This could be caused by any disorder or due to lack of essentials like the glomerular filtration rate (GFR) reduction [5]. Our proposed prediction model takes the clinical symptoms as input and predicts the results using the stacking classifier with the random forest algorithm as a base classifier.

Machine learning is gaining significance in healthcare diagnosis as it enables intricate analysis, thereby minimizing human errors and enhancing the precision of predictions. Machine learning algorithms and classifiers are now considered the most reliable techniques for the diagnosis of different diseases like heart disease, diabetes, tumors disease, and liver disease predictions [6].

Different machine learning algorithms used the Naïve Bayes, SVM, and the decision tree for the classification purpose, while random forest, logistic regression, and linear regression were used for the regression purpose in the medical fields for the prediction. With the efficient use of these algorithms, the death rate can be minimized due to early-stage diagnosis and patients can be treated timely. Along with maintaining the clinical symptoms, chronic kidney disease patients should include physical activities in daily life. They should exercise, drink water, and avoid junk food. The common symptoms of chronic kidney disease are shown in Figure 1.

This article delivers an overview and analysis subsequently followed by an implementation and evaluation of the machine learning classifiers used in CKD diagnosis. Further, this article discusses the importance of machine learning classifiers in healthcare and explains how these can make more accurate predictions.  Figure 2 represents the block diagram of the chronic kidney disease prediction model.

The core objective of this article is to propose and implement a hybrid machine learning prediction model for chronic kidney disease where due importance is given to accuracy. In this article, we have analyzed the accuracy of same dataset with respect to different machine learning algorithms and compared their accuracy score so as to get a better model. Our focus remains on the solution of overfitting problem using cross-validation while achieving the highest accuracy to build a best hybrid model from the combination of available popular machine learning classifiers such as decision tree, gradient boosting, Gaussian Naïve Bayes, and gradient boosting. The ultimate goal is to deliver an accurate and effective treatment to CKD patients at a reduced cost. Before we proceed further, we need to know little more about common diseases of the kidney. In Table 1, there is a list of some of the most common kidney diseases (Table 2).

The remaining portion of the article is organized as follows. Section 2 contains the literature survey along with the tabular comparison of the different machine learning algorithms used and an analysis of the results. Section 3 contains the proposed methodology. Section 4 contains the dataset details. Section 5 contains results and discussion.  Section 6 contains conclusion and future work.

## 2. Literature Review

This section covers research work related to algorithms and assesses some algorithms based on their accuracy. In research work [7], the data mining technique applied to specific analysis of clinical records is a good method. The performance of the decision tree method was 91% (accuracy) compared to the Naïve Bayesian method. The classification algorithm for diabetes dataset had 94% specificity and 95% sensitivity. They also found that mining helps retrieve correlations of attributes that are no longer direct indicators of the type they are trying to predict. Similar work still needs to be done to improve the overall performance of prediction engine accuracy in the statistical analysis of neural networks and clustering algorithms.

In [8], the authors described the prediction models using machine learning techniques including K-nearest neighbor (KNN), support vector machine (SVM), logistic regression (LR), and decision tree classifiers for CKD prediction. From the experiment, it was concluded that the SVM classifier provides the highest accuracy, 98.3%. SVM has the absolute best sensitivity after training and testing performed with the proposed method. Therefore, according to this comparison, it could be concluded that an SVM classifier is used to predict persistent kidney disease.

In the paper [9], they chose four different algorithms and compared them to get an accurate expectation rate over the dataset. Unlike all approaches that were presented, they got the best results from the gradient boosting classifier. The models effectively achieve an accuracy rate of 99.80%, whereas AdaBoost and LDA achieve 97.91% at a low value. Also, the gradient boosting ML classifier takes much time to make the prediction compared to others and has a higher predictable value in both the curves (ROC and AUC). Hence, an accurate expectation undoubtedly depends on the preprocessing strategy, and the methods of preprocessing must be approached cautiously to precisely achieve recognized results.

In [7], the authors investigated the machine learning ability, which is supported by predictive analysis so as to predict CKD early. An experimental procedure was performed by considering a dataset of 400 cases collected by Apollo Hospitals India. In this article, two labels were used as output/targets in this hybrid model (i.e., patients having CKD and others who are healthy) and four different machine learning classifiers were implemented. On the comparison of these classifiers, the classification along with regression tree, and the RPART classification model, showed remarkably better results in terms of accuracy. They used the information gain quotient for excruciating criterion, and here the optimum spilling reduces the noise of the resulting feature subsets. In this study, the RPART limited value of criterion for the splitting was five, meaning that splits repeatedly occur for the five instances present in the leaf node. In addition, they identified an equivalent previous probability for the class attributes. Here, the RPART prediction model used seven terminal nodes for the earlier predictions of CKD. The experimental results showed that the highest AUC and TPR were obtained with the machine learning prediction model, whereas the highest TNR (1.00) was achieved with the model RPART. The RPART model could be described as a set of rules for making the decision. However, the major drawback of RPART is the consideration of the single factor as a parameter in every division procedure, while considering different parameter combinations could result in better CKD predictions. However, the machine learning prediction model gives the lowest error rate. The major reason is that the MLP could adopt and handle complex predictions. The complex relationships require hidden nodes and they are useful as they allow neural networks to model between parameters while sometimes deal with nonlinearity in data. The overall results indicate that the algorithms of machine learning give an inspiring and a feasible methodology for earlier CKD prediction.

As we have already seen, there are different machine learning prediction models and learning programs available to assist practitioners. In [5], they used a new selection guide for predicting CKD. In this work, CKD is predicted by using specific classifiers and a reasonable study of overall performance. In this study, they performed the evaluation of the Naïve Bayes classifier, random forest, and artificial neural network classifiers and concluded that the random forest classifier performs better as compared to other classifiers. The worth of forecasting CKD has been progressive. Several sustainable evolutionary policies can be used to improve the outcomes of the suggested classifiers. Here, Naïve Bayes, random forest, and KNN were applied to predict CKD. Early diagnosis of CKD helps to treat those affected well in time and prevent the disease from progressing to worse stage. The early detection of this type of disease and well-timed treatment is one of the main objectives of the medical field.

In [10], a machine learning prediction model was developed for the early prediction of CKD. The dataset gives input features gathered from the CKD dataset and the models were tested and validated for the given input features. Machine learning decision tree classifier, random forest classifier, and support vector classifier were constructed for the diagnosis of CKD. The performance analysis of the models was assessed on the basis of the accuracy score of the prediction model. On comparison, the results of the research showed that the random forest classifier model performs much better at predicting CKD as compared to decision tree and support vector classifiers.

The kidneys play a vital role in maintaining the body's blood pressure, acid-base sense of balance, and electrolyte sense of balance, not only needed to filter toxins from the body. Malfunction is accountable for insignificant to mortal illnesses, in addition to dysfunction in the other body organs. Therefore, researchers all over the world have dedicated themselves for finding techniques to accurately diagnose and effectively treat chronic kidney disease. As machine learning classifiers are increasingly used in the medical field for diagnosis, now CKD is also included in the list of diseases that could be predicted using machine learning classifiers. The research to detect CKD with ML algorithms has enhanced the procedure and consequence accuracy progressively. They proposed the random forest classifier (99.75% accuracy) as the maximum efficient classifier among all other classifiers. The study demonstrates the effective handling of missing values in data through four techniques, namely, mode, mean, median, and zero-point methods. It also evaluates the performance of machine learning models under two scenarios, with and without tuning the hyperparameters, and observes significant improvement in the classifiers' performance, which is visually presented through graphs [11].

Overall, the motive of the study is to examine the applicability of specific supervised machine learning classifiers in the field of bioinformatics and offer their compatibility in detecting several serious diseases such as the diagnosis of CKD at an early stage [12].

They built an updated and proficient machine learning (ML) application that can perceptually perceive and predict the state of chronic kidney disease. In this work, the ten most important machine learning methods for predicting permanent kidney disease were considered. The level of accuracy of the classification algorithm we used in our project is as good as we wanted.

For the prediction of disease, the first most essential step is to detect the disease that is costly in developing countries like Pakistan and Bangladesh. The people of these countries mostly suffer from this. Currently, CKD patient proportion is increasing rapidly in Pakistan and Bangladesh. So, in that article, the authors tried to develop a system that helps in predicting the risk of CKD. In the proposed model, they used and processed UCI datasets and real-time datasets and tried to deal with missing data and trained the model using random forest and ANN classifiers. Then, they implemented these two algorithms in the Python language. The accuracy they got with the random forest algorithm is 97.12% and that with ANN is 94.5%, which is relatively very good. By use of this proposed method, risk prediction of CKD at an early stage is possible.

In [13], the authors predicted CKD based on sugar levels, aluminum levels, and red blood cell percentage. In this perception, five classifiers were applied, namely, Naïve Bayes, logistic regression, decision table, random tree, and random forest, and for each classifier, the results were noted based on (i) without preprocessing, (ii) SMOTE with resampling, and (iii) class equalizer. Random forest classifier has been observed to give the highest accuracy at 98.93% in SMOTE with resampling.

### 2.1. Comparison of Machine Learning Classifiers for CKD

In this section, a comprehensive comparison of the state of the art is presented in the form of a table. The evaluation is formed in the aspect of accuracy, which can be comprehended in Table 3. The table has eight features that are described below:

  Author: this contains the names of the authors of each article along with the reference.
  Year: this column provides the year of the paper's publication.
  Input data: this column shows the type of dataset that was used as input for the machine learning classifiers.
  Disease type: This section shows the type of disease that was predicted by using different classifiers. It shows the best classifier found in the research paper, which is the classifier with the maximum accuracy.
  Classifiers: this column signifies the different machine learning classifiers that were used in the research and the comparison between them.
  Tool: The column represents the programming language or the framework that was used in building the model. The researchers used these tools to preprocess the input data, then create a prediction model, and finally go to the testing stage.
  Cross-validation: this column gives information about the validation of the classifiers and makes a comparison of different research papers regarding folds of cross-validation used.
  Accuracy: The accuracy of the outcomes of the recommended model is represented in this column. If the article crisscrosses a comparison, the accuracy column only contains the accuracy percent of the best classifier confirmed by the author.

### 2.2. ML Classifier with Highest Accuracy

The machine learning algorithms that we analyzed from the above literature are listed in Table 4 and Figure 3.

## 3. Proposed Methodology

The proposed hybrid model is implemented in Python with pandas, sklearn, Matplotlib, Plotly, and other essential libraries. We have downloaded the CKD dataset from the UCI repository. The dataset contains two groups (CKD represented by 1 and non-CKD represented by 0) of chronic kidney disease in the downloaded information. The machine learning algorithm that has best accuracy is selected for analysis and implementation so that repeated results are produced. We have also developed a hybrid model based on knowledge that we gained during the analysis and implementation. The hybrid model consists of Gaussian Naïve Bayes, gradient boosting, and decision tree as base classifiers and random forest as a meta classifier. We have selected the tree-based machine learning algorithms for achieving the highest accuracy, while at the same time, it can handle the overfitting problem. In this paper, we detect the outliers with the violin plot as shown in Figure 4. As a solution of this problem, we implement the *k*-fold technique and design our model in such a way that it can reduce the problem of overfitting along with achieving the highest accuracy. The classifiers are discussed as under.

### 3.1. Naïve Bayes (NB)

The NB classifier is related to the group of probabilistic classifiers and is constructed on the basis of the Naïve Bayes (NB) theorem. It takes up vigorous independence between the component's/features, and it contains the most crucial part of how this classifier creates forecasts. It can be built easily and is appropriately used in the medical field for the prediction of different diseases [15].

### 3.2. Decision Tree (DT)

The decision tree classifier has a tree-like configuration or flowchart-like construction. It consists of subdivisions, leaves/child nodes, and a root/parent node. Here inner nodes comprise the features, whereas the subdivisions epitomize the outcome of every check on every node. Decision tree is one of the commonly used classifiers for classification determination because it does not need abundant information in the field or place constraints for it to work [15].

### 3.3. Random Forest (RF)

In the ensemble and stacking classification approach, the random forest (RF) is the most effective algorithm among the other machine learning algorithms. In prediction and probability estimations, random forest (RF) algorithm has been used. Random forest (RF) classifier consists of many decision trees. Tin Kam Ho of Bell Labs introduced the concept of random forest in 1995, where each decision tree casts a vote to determine the object's class. The RF method is the combination of both bagging and random selection of attributes. Random forest classifier has the three hyperparameter tuning values [16].

- Number of decision trees (*n* tree) used by the random forest classifier
- Size of the minimum node in the trees
- Number of attributes employed in splitting every node for every tree (*m* try). Here, m is the number of attributes.

Some of the advantages of the random forest classifier are listed as follows.

- For ensemble learning algorithms, the random forest is the most appropriate choice
- For large datasets, random forest classifier performs well
- Random forest (RF) is able to handle hundreds of input attributes
- Random forest can estimate which attributes are more important in classification
- Missing value can be handled by using random forest classifier
- Random forest handles the balancing error for class in unbalanced datasets

### 3.4. Gaussian Naïve Bayes (GNB)

Gaussian Naïve Bayes (GNB) calculated the mean and standard deviation of each attribute at the training stage. To calculate the probabilities for the test data, mean and standard deviation were used. Due to this reason, some values of attributes are too big or too small from the value of the mean calculated. It affects the classifier performance when testing data patterns have those attribute values and gives sometimes wrong output labels [22].

### 3.5. Hybrid Model

We use the concept of stacking for our hybrid model. As a type of ensemble technique in stacking, multiple classification models were combined with a main/meta classifier. One after the other, multiple layers were placed, where the models pass their predictions, and the upper most layer model makes decisions on the base of the combination of different models as a base model. The models in the low layer get attributes as input from the original data. The topmost layer of the model gets output from the lower layers and gives the results as a final prediction. The stacking technique involves using multiple independent machine-learning models as input to process the original data. After that, the meta classifier is used to predict the input along with the output of each machine learning model and individual algorithm's weights are estimated. The algorithms that are performing best are selected, and others having low performance are removed. In this technique, multiple classifiers as base model are combined and then, by using different machine learning algorithms, are trained on the same dataset through the use of a meta-classifier [23].  Figure 5 shows the flow diagram for the proposed hybrid model.

The execution of the model with the sequence of the steps is given below:

- Collect the data of CKD from UCI repository
- Exploratory data analysis (EDA) is performed on that dataset
- This dataset is split into two parts: test data and train data
- Apply the cross-validation of 10 folds
- Train the base models Gaussian Naïve Bayes, gradient boosting, and decision tree with the train set giving the predictions as M1, M2, and M3, respectively
- The output of the base models M1, M2, and M3 and test set data serve as input for random forest as input for training
- Once the random forest gets trained, it gives the prediction on the basis of training dataset and the output predictions of the base models

In this study, we have considered the UCI CKD dataset, and this dataset is split into two parts. 80% of data is used for training purposes as an input to the machine learning algorithms. We exploited the Gaussian Naïve Bayes, gradient boosting, decision tree, and stacking classifier with random forest algorithm which was used to predict the chronic kidney disease for 20% test data as input and plotted the predicted values and compared their values. Our proposed methodology has the following advantages.

- We implemented four machine learning algorithms that are decision tree, gradient boosting, Gaussian Naïve Bayes, and random forest. We applied stacking classifiers to build the hybrid model that combines these four algorithms.
- We analyzed the accuracy of the same dataset with respect to different machine learning algorithms and compared their accuracy score to get the best model
- We implemented a stacking classifier technique to build a new model with improved accuracy

## 4. Dataset Details

We selected 14 attributes from the dataset that we are using from the UCI repository dataset of chronic kidney disease as input features as shown in Table 5 where age attribute shows the patient's age, bp indicates the blood pressure, sg indicates the specific gravity of the urine, al indicates the level of aluminum in the patient urine, bgr (blood glucose random) indicates the blood sugar level glucose tolerance, su represents the sugar level, bu indicates the blood urea, sod indicates the amount of sodium, sc indicates the serum creatinine, pot indicates the amount of potassium, hemo indicates the hemoglobin, and pcv indicates the packed cell volume. Further, wc indicates the white blood cell count, and rc indicates the red blood cell count.

To identify the number of chronic kidney disease patients and the number of healthy ones, we performed the visualization on the CKD dataset, which can be seen in the histogram plot in Figure 6. Here 0.0 represents the healthy cases, while 1.0 represents the chronic kidney disease patients. In this dataset, there are 250 chronic kidney disease patients, while 150 are healthy people.

The Pearson correlation feature selection method is used to get the best combination of features for the prediction of chronic kidney disease. The correlation of the 14 attributes and 1 output label is presented in Figure 7.

When we go from the exploratory data analysis stage to the pair plot visualization, it is observed to be very helpful as it gives the data that can be used to find the relationship between attributes for both the categorical and continuous variables. We import the Seaborn library to get pair plot. The information about all the attributes is in one picture and is clear. The statistical information is in attractive format represented with pair plot as shown in Figure 8.

The violin plots are used for all the attributes in exploratory data analysis that are used in the hybrid model. These can give additional useful information like density trace and distribution of the dataset. The violin plots give the whole range of dataset which cannot be shown by box plot. The violin plots of all 14 attributes are given in Figure 4.  Figure 9 shows the comparison of different models' accuracy scores in the form of a chart.

## 5. Results and Discussion

Machine learning algorithms such as gradient boosting, Gaussian Naïve Bayes, decision tree, and random forest classifier were used in the proposed hybrid model. These different machine learning classifiers were used as a combination for the chronic kidney disease predictions. This also overcomes the overfitting problem and results in higher accuracy. In order to improve accuracy and to come up with a novel approach as compared to the existing work, we have implemented the proposed hybrid model with the best combination of GB, GNB, and decision tree, along with the random forest classifiers [24–27]. The results described in Table 6 show that diagnosis of chronic kidney disease is effective using the random forest with combination as a stacking technique in the hybrid model. Gradient boosting achieves 99% accuracy, random forest achieves 98% accuracy, and our hybrid model achieves 100% accuracy, and at the same time, it has reduced the chances of overfitting.

In order to find the contributions to the development of prediction models for chronic kidney disease, a regional basis analysis is performed. As discussed in the Introduction section that the developing countries' population suffers more from chronic kidney disease, it was observed that most of the research work is performed in developing countries. A summary of this region-wise contribution is presented in Figure 10.

## 6. Conclusion

Chronic kidney disease is considered as one of the prominent life-threatening diseases in the developing world. The most obvious cause seems to be lack of physical exercise. The medical practitioners used a number of diagnosis processes and procedures, where machine learning is the recent development. In this paper, we have selected machine learning because in terms of accuracy, it performs better as compared to other available approaches. In this article, we have used the Pearson correlation feature selection method and applied the same on machine learning classifier. GB, GNB, decision tree, and random forest are the base classifiers for the stacking algorithm, whereas these are implemented with the cross-validation on the basis of accuracy score. In this study, we evaluated these algorithms on the same dataset. Furthermore, we have used dataset of CKD from the UCI directory that contains 14 attributes and 400 instances. On the basis of these attributes, our proposed stacking model is able to predict whether the person is a CKD patient or not with 100% accuracy. Best features are selected using the Pearson correlation method, and the stacking algorithm is implemented with the best machine learning classifiers. The cross-validation enhances the performance of the stacking model. As we have worked on the chronic kidney disease data of the binary group, the stacking algorithm performs better with these combinations of algorithms. We can implement the stacking technique for the prediction of other diseases to get better accuracy score.

## Figures and Tables

**Figure 1:** Symptoms in CKD patients [7].

**Figure 2:** Block diagram of the machine learning hybrid model.

**Figure 3:** Comparison of machine learning classifiers.

**Figure 4:** Violin plot of attributes.

**Figure 5:** Flowchart for the proposed model.

**Figure 6:** Histogram plot.

**Figure 7:** Heat map of chosen attributes.

**Figure 8:** Pair plot of each attribute.

**Figure 9:** Accuracy score of implemented machine learning classifiers.

**Figure 10:** Region-wise contributions.

**Table 1:** Description of common diseases of the kidney.

Diseases	Description
CKD	Chronic kidney disease (CKD) can occur when a disease or condition damages kidney function, causing kidney damage to deteriorate over a few months or years.
Kidney stones	Kidney stones (also called renal calculi) are hard pledges made of salts and minerals that form inside your kidney.
Glomerulonephritis	Glomerulonephritis causes infection and damage to the filtering part of the kidneys (glomerulus). It can occur quickly or could be over a longer period. Poisons, metabolic wastes, and surplus fluid are not properly strained into the urine. Instead, they build up in the body producing inflammation and fatigue.
Polycystic kidney disease	Polycystic kidney disease (PKD) is a genetic disorder that can produce many cysts filled with fluid and they grow inside your kidneys. Usually, they are harmless. The cysts can change the shape of the kidneys while making them much bigger.

**Table 2:** Equations for accuracy measurement.

S. no	Authors	Accuracy equations
1	Padmanaban and Parthiban [8]	Precision *i* = TPi/TPi + FPi
2	Charleonnan et al. [9]	ACC = (TP + TN)/(P + N)
3	Ghosh et al. [7]	The results of performance degree indices are dependent on TP, TN, FP, and FN
4	Fu et al. [10]	Ext. values = points > Q3 + 1.5 (IQR) points < Q1 − 1.5 (IQR)
5	Devika et al. [11]	Accuracy = number of properly classified samples/total variety of samples
6	Revathy et al. [12]	Accuracy =(TP+TN)/(TP+TN+FP+FN) Accuracy = TP + TN/TP + TN + FP + FN
7	Nishat et al. [14]	Accuracy =(TP+TN)/(TP+TN+FP+FN) Accuracy = TP + TN/TP + TN + FP + FN
8	Rabby et al. [13]	Descriptive analysis of the data as well as the experimental results
9	Pouriyeh et al. [15]	Finding most significant feature using chi-square test
10	Jabbar et al. [16]	Experimental results only

True positive (TP) = list contains stated cases that are correctly categorized with CKD. False positive (FP) = list contains set that is inaccurately categorized with CKD. True negative (TN) = list contains stated instances that are correctly categorized with CKD. False negative (FN) = list contains set of instances that are exactly categorized with CKD.

**Table 3:** Comparison of classifiers for CKD.

S. no	Authors	Year	Input data	Disease type	Tools	Classifiers	Cross-validation	Accuracy
1	Padmanaban and Parthiban [8]	2016	Diabetic patients	CKD	WEKA, YALE	Naïve Bayes	10 folds	86%
			UCI machine learning			Decision tree		**91%**

2	Charleonnan et al. [9]	2016	Clinical data	CKD	WEKA, MATLAB	SVM	5 folds	**98.3%**
						Logistic regression		96.55%
						Decision tree		94.81%
						KNN		98.1%

3	Ghosh et al. [7]	2020	Apollo Hospitals India	CKD	Python	SVM	5 folds	99.56%
						AB		97.91%
						LDA		97.91%
						GB		**99.80%**

4	Fu et al.. [10]	2018	UCI repository (CKD dataset)	CKD	Python	RPART	No cross-validation	98.2%
						SVM		97.3%
						LOGR		99.4%
						MLP		**99.5%**

5	Devika et al. [11]	2019	UCI repository (CKD dataset)	Chronic renal disorder	C Sharp	Naïve Bayes	No cross-validation	99.63%
						KNN		87.78%
						Random forest		**99.84%**

6	Revathy et al. [12]	2019	UCI repository (CKD dataset)	CKD	Python	Decision tree	No cross-validation	94.16%
						SVM		98.33%
						Random forest		**99.16%**

7	Nishat et al. [14]	2021	Learning repository of University of California, Irvine	CKD	Python	CNN	No cross-validation	78%
						LR		98.25%
						DT		99%
						RF		**99.75%**
						SVM		85%
						NB		96.5%
						MLP		81.25%
						QDA		37.5%

8	Rabby et al. [13]	2019	UCI repository (CKD dataset)	CKD	Python	K-nearest neighbor	No cross-validation	71.25%
						RF		98.75%
						SVM		97.50
						GNB		**100%**
						AB		98.75%
						DT		**100%**
						LDA		97.50%
						GB		98.75
						LR		97.50%
						ANN		65%

9	Pouriyeh et al. [15]	2020	UCI repository (CKD dataset)	CKD	Python	RF	10 folds	**97.12%**
						ANN		94.5%

10	Jabber et al. [16]	2020	UCI repository (CKD dataset)	CKD	Python	Decision tree	No cross-validation	96.79%
						Logistic regression		97.86%
						Naïve Bayes		97.33%
						Random forest		**98.93%**

11	Bmc [17]	2013	UCI repository	Diabetic kidney disease	MATLAB	SVM	No cross-validation	0.91
						PLS		0.83
						FFNN		0.85
						RPART		0.87
						Random forest		**0.91**
						Naïve Bayes		0.86
						C5.0		0.90

12	Ramya and Radha [18]	2016	UCI repository	Chronic kidney disease	R	BP	No cross-validation	80.4
						RBF		85.3
						Random forest (RF)		78.6

13	Kumar [19]	2016	UCI repository	CKD	MATLAB	RF	No cross-validation	95.67
						SMO		90
						Naïve Bayes		87.64
						RBF		83.78
						MLPC		89
						SLG		87

14	Basarslan and Kayaalp [20]	2019	UCI repository	Chronic kidney disease	MATLAB	K-nearest neighbor	No cross-validation	97
						Naïve Bayes		96.5
						LR		97.56
						RF		99

**15**	Dowluru and Rayavarapu [21]	2012	UCI repository	Kidney stone	WEKA tool	Naïve Bayes classification	No cross-validation	0.99
						Logistic regression		1.00
						J48 algorithm		0.97
						Random forest		0.98
					Orange tool	Naïve Bayes		0.79
						KNN		0.7377
						Classification tree		0.9352
						C4.5		0.9352
						SVM		0.9198
						Random forest		0.9352

Bold values represent the highest accuracy in the relevant paper.

**Table 4:** Machine learning algorithms and classifiers.

Articles	Classifiers	Highest accuracy (%)
1	Decision tree	91

2	SVM	98.3

3	GB	99.80

4	MLP	99.5

5	Random forest	**99.84**

6	Random forest	99.16

7	Random forest	99.75

8	GNB	**100**
	Decision tree	**100**

9	Random forest	97.12

10	Random forest	98.93

Bold values represent the highest accuracy in the literature.

**Table 5:** The attribute set with their data types.

#	Attributes	Full form	Data type	Nonempty value	Missing values
0	age	Age	float64	400	0
1	bp	Blood pressure	float64	400	0
2	sg	Specific gravity of urine	float64	400	0
3	al	Level of aluminum	float64	400	0
4	su	Sugar level	float64	400	0
5	bgr	Blood glucose random	float64	400	0
6	bu	Blood urea	float64	400	0
7	sc	Sugar level	float64	400	0
8	sod	Amount of sodium	float64	400	0
9	pot	Amount of potassium	float64	400	0
10	hemo	Hemoglobin	float64	400	0
11	pcv	Packed cell volume	float64	400	0
12	wc	White cell	float64	400	0
13	rc	Red cell	float64	400	0

**Table 6:** Accuracy score of implemented machine learning classifiers.

ML algorithms	Accuracy (%)
Gradient boosting	99
Gaussian Naïve Bayes	93
Decision tree	96
Random forest	98
Hybrid model	100

## Data Availability

No data were used to support this study.
